# Involvement of Sex Hormones and Their Receptors in the Pathogenesis of Classic Kaposi's Sarcoma in Xinjiang

**DOI:** 10.1111/srt.70086

**Published:** 2024-09-30

**Authors:** Meng Wei, Xin Jiang, Yi Bian, Jun‐Wei Fan

**Affiliations:** ^1^ Department of Cardiac Pacing and Electrical Engineering the First Affiliated Hospital of Xinjiang Medical University Urumqi China; ^2^ Department of Dermatology The First Affiliated Hospital of Xinjiang Medical University Urumqi China

**Keywords:** androgen receptor, classic Kaposi sarcoma, estradiol, estrogen receptor, pyogenic granuloma, testosterone

## Abstract

**Objective:**

This study aims to examine the expression of androgen receptor (AR) and estrogen receptor (ER) in patients with classic Kaposi's sarcoma (CKS) in Xinjiang, as well as to assess the serum levels of sex hormones in these patients. The objective is to explore potential new directions and targets for diagnosing and treating CKS in Xinjiang.

**Methods:**

The case group comprised 35 patients diagnosed with CKS who presented at our hospital from 2014 to 2021. The control group consisted of 35 patients with pyogenic granuloma (PG) who visited the hospital during the same period, selected using propensity score matching (PSM). Immunohistochemistry was used to detect AR, human herpesvirus type 8 (HHV‐8), and ER in paraffin‐embedded tissue samples from patients diagnosed with CKS and PG. Additionally, enzyme‐linked immunosorbent assay (ELISA) was used to quantitatively measure serum sex hormone levels in the 35 patients with CKS and 35 patients with PG.

**Results:**

AR expression was relatively weak in both the CKS and PG groups, with the PG group exhibiting a slightly stronger expression than the CKS group. Conversely, the expression of ER was significantly higher in the CKS group compared to the PG group (*p* < 0.05). Additionally, serum testosterone (*T*) levels were elevated in the CKS group, while serum estradiol (E2) levels were higher in the PG group (*p* < 0.05).

**Conclusion:**

Sex hormones and their receptors are implicated in the pathogenesis of CKS in Xinjiang. The use of ER antagonists may represent a novel avenue for research and treatment of CKS.

**Abbreviations**
AR: androgen receptor
CKS: classic Kaposi's sarcoma
ELISA: enzyme‐linked immunosorbent assay
ER: estrogen receptor
KS: Kaposi's sarcoma
KSHV: Kaposi's sarcoma‐associated herpesvirus
PSM: propensity score matching

## 1 Introduction

Kaposi's sarcoma (KS) is a mesenchymal tumor, currently believed to originate from lymphatic endothelial cells [1]. This malignancy primarily affects the skin and mucous membranes but can also involve the lymphatic system and internal organs like the gastrointestinal tract, lungs, and liver [2]. Initially, KS was strongly associated with human herpesvirus type 8 (HHV‐8), also known as Kaposi's sarcoma‐associated herpesvirus (KSHV), and annually, over 20 000 patients succumb to this disease [3]. In recent decades, there has been a rising incidence of KS among patients with AIDS and organ transplant recipients. However, in Xinjiang, such patients are relatively rare, and most clinically observed patients have not been infected with the AIDS virus nor have they undergone organ transplantation.

Currently, more than 90% of KS cases in China are reported in Xinjiang. Clinically, KS manifests as purplish‐red papules, plaques, or nodules, predominantly on the extremities. These skin lesions may ulcerate, cause pain, and become secondarily infected, significantly impacting the physical health and quality of life of the patient. The incidence of classical Kaposi's sarcoma (CKS) in Xinjiang primarily affects Uyghur males, indicating a certain ethnic susceptibility. Foreign studies have reported a male‐to‐female ratio of 10:1 for CKS, while our previous research in Xinjiang found a ratio of 7:1, indicating a notable gender difference [4, 5]. Although infection with HHV‐8 is a common cause of all types of KS, the global prevalence of HHV‐8 infection is much higher than the incidence of KS [6, 7]. Therefore, HHV‐8 infection alone cannot account for the observed ethnic and gender disparities in the incidence of KS, nor can ethnic susceptibility fully explain the gender differences among Uyghur patients with KS.

Based on the aforementioned observations, it is hypothesized that sex hormones and their receptors play a crucial role in the pathogenesis of CKS in Xinjiang. The objective of this study is to compare CKS with patients diagnosed with pyogenic granuloma (PG), as PG is also a vascular‐origin tumor characterized by vascular endothelial hyperplasia, tumor collapse, and bleeding, both pathologically and clinically. Immunohistochemistry was used to detect the expression of androgen receptor (AR) and estrogen receptor (ER) in the pathological tissues of patients diagnosed with CKS and PG. Additionally, serum levels of estrogen and androgen in both patient groups were measured. The goal was to examine the underlying reasons for the significant gender disparity among patients diagnosed with CKS in Xinjiang and to explore new directions and targets for the diagnosis and treatment of CKS in Xinjiang.

## 2 Materials and Methods

### 2.1 Selection of Case Group and Control Group

In this study, 35 paraffin‐embedded tissue blocks diagnosed as CKS using clinical, pathological, and immunohistochemical methods at the First Affiliated Hospital of Xinjiang Medical University between 2014 and 2021 were selected as the case group. Blood samples from these patients were extracted and stored in a refrigerator at −80°C. The inclusion criteria were as follows: (1) patients with CKS which was diagnosed both clinically and pathologically; (2) tumor stage pathology; (3) positive immunohistochemical staining for HHV‐8; (4) signed informed consent forms and approval by the Ethics Committee (approval ID: 20190905−17). Exclusion criteria was: (1) patients not registered in Xinjiang or foreigners; (2) patients with AIDS or suspicious/positive HIV test results; (3) patients with a history of kidney, bone marrow, or other organ transplants; (4) cases where skin pathology application forms had defects or other issues preventing satisfactory clinical data collection; (5) pregnant women or other special cases. The control group consisted of 35 patients with PG, with paraffin‐embedded tissues collected during the same period as the CKS group. Propensity score matching (PSM) with a 1:1 ratio was used to ensure that the baseline data of both groups were balanced.

### 2.2 Experimental Reagents, Consumables, and Instruments

The details of the specific experimental instruments, consumables, and reagents are provided in Table 1.

**TABLE 1:** Specific information on instruments, reagents, and consumables.

Reagents/consumables	Manufacturer	Article no.
PBS	Fuzhou Maxin Biotechnology Development Co., Ltd	PBS‐0060/0061
Citric acid powder	Fuzhou Maxin Biotechnology Development Co., Ltd	MVS‐0066
Immunohistochemical staining kit	Beijing Zhongshan Jinqiao Biotechnology Co., Ltd	SP9000
Hematoxylin stain	Fuzhou Maxin Biotechnology Development Co., Ltd	CTS‐1097
DAB color reagent kit	Fuzhou Maxin Biotechnology Development Co., Ltd	DAB‐1031
Antibody diluent	Beijing Zhongshan Jinqiao Biotechnology Co., Ltd	ZLI‐9029
neutral balsam	Beijing Zhongshan Jinqiao Biotechnology Co., Ltd	ZLI‐9555
Rabbit anti‐androgen receptor antibody	Beijing Boaosen Biotechnology Co., Ltd	bs‐0118R
Rabbit anti‐estrogen receptor alpha antibody	Beijing Boaosen Biotechnology Co., Ltd	bs‐0725R
Rabbit anti‐HHV8 ORF50 antibody	Beijing Boaosen Biotechnology Co., Ltd	bs‐0859R
Microplate reader	Bio‐Rad	xMark
Electric thermostatic incubator	Shanghai Jinghong Test Equipment Co., Ltd	DNP‐9272
Micro oscillator	Jintan Medical Instrument Factory	MM‐2
Human E2 ELISA Kit	Wuhan Huamei Bioengineering Co., Ltd	CSB‐E05108h
Human testosterone ELISA Kit	Wuhan Huamei Bioengineering Co., Ltd	CSB‐E05099h
Constant temperature blast drying oven	Shanghai Jinghong Experimental Equipment Co., Ltd	DHG Type
Refrigerator	Hefei Meiling Co., Ltd	BCD‐249LCK
Pressure cooker	Zhejiang Supor Co., Ltd	YW20F1
Electromagnetic furnace	Guangdong Midea Life Appliance Manufacturing Co., Ltd	C21‐RK2101
Microscope	Nikon biological microscope	E200

Abbreviations: E2, estradiol; PBS, phosphate buffer solution.

### 2.3 Preparation of Experimental Reagents

1. PBS (pH 7.4–7.6): A bag of PBS powder was dissolved in 2000 mL of distilled water, stirred until the powder was fully dissolved, and mixed thoroughly to prepare the working solution. The solution was kept at room temperature for use.
2. Powder Antigen Repair Solution (citric acid method): The powder antigen repair solution was dissolved from the bags in 2000 mL of distilled water to prepare the working solution.
3. Gradient Ethanol (100%, 95%, 90%, 80%, 70%): The gradient dilution of anhydrous ethanol was prepared with distilled water.
4. 3% H₂O₂ Solution: The researchers mixed 50 mL of 30% H₂O₂ with 450 mL of distilled water to prepare the solution (ready for use).
5. 1% Hydrochloric Acid Alcohol Differentiation Solution: Concentrated hydrochloric acid was combined with 75% alcohol in a ratio of 1:99.
6. DAB Chromogenic Agent: In a 1.5 mL centrifuge tube, 0.85 mL of distilled water was added. Sequentially 50 µL each of reagents A, B, and C were added and were mixed well after each addition to prepare 1 mL of DAB color‐developing solution. This had to be prepared on the spot and stored away from light.
7. ELISA (enzyme‐linked immunosorbent assay) Reagents: Provided by the kit.

### 2.4 Immunohistochemical and ELISA

The tests were conducted following the standard procedures outlined in the kit. After completing the immunohistochemistry, the staining intensity and percentage of stained cells were assessed and scored, with subsequent analysis performed on images captured under the microscope.

### 2.5 Statistical Methods

The data for this study were analyzed using SPSS version 23.0 (IBM Corp., Chicago, IL, USA). Continuous variables in the baseline data were described using mean ± standard deviation (SD). For normally distributed data with uniform variance between groups, a two‐independent‐samples *t*‐test was used. Immunohistochemical scores, which did not follow a normal distribution, were analyzed using the rank sum test on the total score derived from the product of two scores. Counting data were expressed as percentages, and comparisons between groups were made using the chi‐square test. The significance level for statistical tests was set at *α* = 0.05.

## 3 Results

### 3.1 Comparison of Baseline Data Between CKS Group and PG Group

The comparison of baseline data between the CKS group and the PG group revealed no significant differences in age, gender, nationality, duration of disease, or distribution of skin lesions (*p* > 0.05). These results indicate that the two groups are comparable with respect to these confounding factors (Table 2).

**TABLE 2:** Comparison of baseline data between the CKS group and PG group (Mean ± SD,%).

Characteristics	CKS group	PG group	*χ*2/*t*	*p*
Age	59.93 ± 12.48	56.25 ± 15.37	1.100	0.275
Gender				
Male	30 (85.71)	28 (80.00)	0.402	0.526
Female	5 (14.29)	7 (20.00)		
Nation				
Uygur	28 (80.00)	23 (54.29)	1.806	0.179
Other	7 (20.00)	12 (45.71)		
Course of disease				
< 1year	12 (34.29)	17 (48.57)	4.494	0.106
1–5years	15 (42.86)	16 (45.71)		
> 5years	8 (22.85)	2 (5.71)		
Distribution of skin lesions				
Feet	20 (57.14)	4 (11.43)	16.232	< 0.001
Legs	13 (37.14)	3 (8.57)	8.102	0.004
Hands	10 (28.57)	9 (25.71)	0.072	0.788
Upper limb	9 (25.71)	3 (8.57)	3.621	0.057
Trunk	7 (20.00)	4 (11.43)	0.971	0.324
Maxillofacial neck	4 (11.43)	14 (40.00)	7.479	0.006

### 3.2 Comparison of the Expression Levels of *T* and E2 in Plasma of Patients in CKS Group and PG Group

Compared to the PG group, the expression of *T* in the CKS group was significantly higher, whereas the expression of estradiol (E2) was significantly lower (*p* < 0.05) (Table 3).

**TABLE 3:** Comparison of *T* and E2 in plasma between the CKS group and PG group (Mean ± SD).

Index	CKS group	PG group	*t*	*p*
T (ng/mL)	2.47 ± 1.14	0.67 ± 0.31	9.014	< 0.001
E2 (pg/mL)	43.79 ± 15.03	79.87 ± 17.38	−9.29	< 0.001

### 3.3 Expression of AR in Tissue Sections of Patients With CKS and PG

Microscopic observation at magnifications of 40×, 100×, 200×, and 400× revealed that AR protein expression was almost undetectable in the tumor tissues of the CKS group. In contrast, weak AR protein expression was observed in some dermal tissues of the PG group. Both the CKS and PG groups demonstrated strong AR protein expression in the basal layer of certain epidermal regions and in sebaceous gland tissue within the dermis (Figure 1).

**FIGURE 1:** The CKS group had significantly lower AR expression than the PG group. Under a light microscope, Kaposi sarcoma pathology is characterized by hyperplastic vascular cavities and fissures with irregular branches and reticulation in the dermis, as well as spindle cells that fuse into nodules. The image reveals brownish‐yellow granules or cellular structures inside and outside the lumen‐like structures, which are red cells rather than tumor cells. CKS indicates classic Kaposi's sarcoma; PG, pyogenic granuloma.

### 3.4 Expression of HHV‐8 in Tissue Sections of Patients With CKS and PG

Microscopic observation at magnifications of 40×, 100×, 200×, and 400× revealed strong positive expression of HHV‐8 protein in KS tissues of the CKS group. In contrast, the positive expression of HHV‐8 protein in dermal tissues of the PG group was extremely weak, with some tissues revealing almost no detectable expression (Figure 2).

**FIGURE 2:** The expression of HHV‐8 in the CKS group was significantly higher than in the PG group. CKS indicates classic Kaposi's sarcoma; PG, pyogenic granuloma.

### 3.5 Expression of ER in Tissue Sections of Patients With CKS and PG

Microscopic observation at magnifications of 40×, 100×, 200×, and 400× revealed strong positive expression of ER protein in KS tissues of the CKS group. In contrast, the positive expression of ER protein in dermal tissues of the PG group was weak (Figure 3).

**FIGURE 3:** The CKS group had higher levels of ER expression than the PG group. CKS indicates classic Kaposi's sarcoma; PG, pyogenic granuloma.

### 3.6 Immunohistochemical Scoring Results of AR, ER, and HHV‐8 in CKS Group and PG Group

Compared to the PG group, the CKS group exhibited lower expression levels of AR and higher expression levels of ER and HHV‐8 (*p* < 0.05) (Table 4).

**TABLE 4:** Analysis of protein scores in the two groups (Mean ± SD).

Index	CKS group	PG group	*t*	*p*
AR	0.46 ± 0.27	1.07 ± 0.38	−7.742	< 0.001
ER	6.57 ± 1.82	4.63 ± 1.41	4.985	< 0.001
HHV‐8	4.07 ± 1.26	1.13 ± 0.43	13.064	< 0.001

## 4 Discussion

In 1872, Moritz Kaposi, a Hungarian dermatologist, first reported KS, subsequently leading to its global recognition. Other authors later described and named this tumor, which shares identical histological characteristics but is associated with distinct racial and population groups. Based on these observations, KS is categorized into four types: classical, endemic, transplant‐related, and AIDS‐related [8]. CKS predominantly affects older patients in Eastern Europe and the Mediterranean region, with a male‐to‐female incidence ratio of approximately 15:1 [9]. Clinically, it presents as purplish‐blue or reddish‐brown plaques or nodules primarily located on the extremities. Over several years or decades, these lesions may gradually extend to other areas. Approximately 10% of patients may experience involvement of internal organs or oral mucosa.

Initially, untreated lesions appear as erythema or plaques, which can progress to nodules that eventually merge into larger patches. Lymphedema may occur either before or after the appearance of skin lesions. Histologically, CKS is characterized by spindle‐shaped tumor cell infiltration around dilated vessels, accompanied by erythrocyte extravasation, hemosiderin deposition, and fibrosis. The results of this study indicate that patients diagnosed with CKS are predominantly male, with a significant increase in ER expression. This finding may offer new directions or insights for future treatment strategies for CKS.

In China, CKS predominantly affects ethnic minorities in Xinjiang, with a higher incidence among Uyghurs and Kazaks, particularly Uyghurs. The pathogenesis of CKS remains largely unresolved, and treatment options are challenging. For localized cases of classic Kaposi's sarcoma (CKS), surgical resection is the primary approach. However, many patients present with multiple skin lesions, significant pain, and a tendency for ulceration and secondary infection, which causes considerable discomfort. For disseminated cases of CKS, traditional treatments primarily include radiotherapy and chemotherapy. Despite the use of radiotherapy, chemotherapy, combination therapies, or interferon treatments, these approaches often exhibit slow efficacy, inability to achieve complete eradication, and significant side effects, along with high costs [10]. Consequently, there is a need for the development and exploration of new, more effective treatment methods for KS.

Currently, extensive research on sex hormone levels and their receptor expression in KS is limited. Our findings indicate that in patients with CKS, predominantly males, serum testosterone levels are elevated compared to healthy patients, whereas serum E2 levels are lower. Additionally, our study found minimal expression of AR in tissue samples from patients diagnosed with CKS. In contrast, ER was positively expressed in both PG and CKS tissues. Notably, the immunohistochemical scores for ER were significantly higher in CKS cases than in the PG group, which was contrary to our initial clinical expectations.

These findings underscore the complex interactions between sex hormones and their receptors in the pathology of CKS. Further detailed investigations are needed to clarify the mechanisms driving these changes in hormone levels and receptor expressions in CKS. Gaining a deeper understanding of the roles of sex hormones and their receptors in CKS is crucial, as it may lead to innovative strategies for treatment and prevention. This highlights the necessity for continued research to enhance our knowledge and enhance patient outcomes.

Although CKS is currently classified as a tumor of lymphatic endothelial origin, histopathological examination reveals spindle‐shaped vessel proliferation and erythrocyte extravasation. Immunohistochemical analysis reveals strong positivity for CD31 and CD34, indicating a significant association with vascular endothelial cells [3]. Our experimental results indicate that ER is closely linked to vascular tumors. Research indicates that abnormalities in ER signaling pathways are associated with the development and progression of various cancers, including breast cancer, ovarian cancer, prostate cancer, and colon cancer [11, 12]. Additionally, foreign studies have indicated that ER, located outside the nucleus, activates rapid‐response molecules like SRC and PI3K/AKT, thereby enhancing the tumorigenic potential of prostate cancer cells and increasing cell proliferation, migration, invasion, and tumor formation [13, 14, 15].

## 5 Conclusion

In conclusion, we hypothesize that ER may play a role in the development of KS. Currently, immunohistochemistry for HHV‐8 is considered the gold standard for diagnosing KS; however, ER immunohistochemistry could provide additional diagnostic value for KS. Furthermore, the strong positive expression of ER in CKS tissues indicates potential therapeutic applications, like using ER antagonists as a treatment target in future clinical research. However, existing studies are insufficiently comprehensive, and further research is needed to elucidate the specific mechanisms by which sex hormone levels and receptors influence CKS. These findings not only enhance the understanding of CKS pathogenesis but also offer new perspectives for the treatment and prevention of related conditions. Longitudinal studies are essential to clarify the underlying causes of these phenomena. Therefore, examining sex hormone levels and receptor expression in CKS is of significant clinical and scientific importance, potentially paving the way for innovative diagnostic and therapeutic strategies.

## Ethics Statement

The present research was approved by the Ethical Committee of the First Affiliated Hospital of Xinjiang Medical University (Approval ID: 20190905–17). This study was conducted in accordance with the declaration of Helsinki.

## Consent

In this study, we were permitted to collect the blood samples and pathological tissue of related patients to detect the biochemical parameters. Written informed consent was obtained from all participants.

## Conflicts of Interest

The authors declare no conflicts of interest.

## Data Availability

The datasets used or analyzed during the current study are available from the corresponding author upon reasonable request.
